The article "Evaluation of Dentinal Microcracks following Diode Laser- and Ultrasonic-Activated Removal of Bioceramic Material during Root Canal Retreatment" was published in 2022. Journal: Scanning.

# Evaluation of Dentinal Microcracks following Diode Laser- and Ultrasonic-Activated Removal of Bioceramic Material during Root Canal Retreatment

**DOI:** 10.1155/2022/6319743

**Published:** 2022-11-21

**Authors:** Reem M. Barakat, Rahaf A. Almohareb, Aljuharh Alsayyar, Fayruz Almalki, Hissah Alharbi

**Affiliations:** ^1^Department of Clinical Dental Sciences, College of Dentistry, Princess Nourah Bint Abdulrahman University, P.O. Box 84428, Riyadh 11671, Saudi Arabia; ^2^Dental Intern, College of Dentistry, Princess Nourah Bint Abdulrahman University, P.O. Box 84428, Riyadh 11671, Saudi Arabia

## Abstract

This study is aimed at evaluating the use of microcomputed tomography (micro-CT) analysis and the dentinal microcrack formation following retreatment of bioceramic sealer employing adjunct laser-activated irrigation and ultrasonic-activated irrigation. Thirty sound human single-canal teeth (*n* = 30) obturated using the single-cone technique with bioceramic sealer were retreated using nickel-titanium (NiTi) rotary files. The sample was randomly divided into three equal groups: group 1, the control group, was not subjected to further treatment; group 2 underwent ultrasonic activation of irrigants; group 3 underwent active irrigation with a diode laser (980 nm wavelength). Using micro-CT, the teeth were scanned before and after retreatment protocols. Two calibrated experienced observers viewed the cross-sectional images and calculated the number of dentinal defects. The presence of any crack or craze line on the external root surface or internal canal wall was counted. Data were analyzed using Friedman's two-way analysis of variance and Fisher's exact test. Statistical significance was set at *p* < 0.05. A significant increase occurred in the number of cracks post retreatment protocols, specifically in the coronal and middle canal thirds, compared to pre- and postinstrumentation (*p* = 0.0001). However, ultrasonic- or laser-activated irrigation did not result in a significant increase in the number of cracks (*p* = 0.345). NiTi rotary root canal retreatment was associated with a significant increase in dentinal microcracks. However, employing ultrasonic- or laser-activated irrigation as adjunct retreatment techniques did not reveal a significant increase in dentinal microcracks within the roots.

## 1. Introduction

The primary objective of nonsurgical root canal retreatment is to optimize the removal of all filling materials, bacteria, and debris by thorough cleaning and reshaping [1]. This method, which involves extra mechanical manipulation and root canal preparation, will degrade the root canal dentine's structure and make it more vulnerable to fracture development [2]. As a result of the increased instrument–canal wall contact, a buildup of stress in the dentin leads to the formation of microcracks, which may ultimately lead to fractures and tooth loss [3, 4]. Although weaker dentin caused by retreatment is not always the primary cause of problems, several extrinsic variables, including stress, temperature change, and instrument friction with the root canal wall, all contribute to canal wall deterioration. Additionally, the effect of some sealers, such as bioceramic (BC), may result in the formation of dentine crack defects [2].

The article "Evaluation of Dentinal Microcracks following Diode Laser- and Ultrasonic-Activated Removal of Bioceramic Material during Root Canal Retreatment" was published in 2022. Journal: Scanning.

BC root canal fillings are a feasible alternative to the current gold standard. Researchers have studied BC sealers in depth, and they have shown bioactive, nontoxic, and biocompatible properties [5], in addition to higher binding strength in comparison to other sealers [6]. However, in the event of retreatment, BC has shown more complexity than conventional sealers [7]. Additionally, the effect of removing BC from the root canal system during retreatment is a cause for concern [8].

In clinical practice, no scientifically proven methods exist for removing BC sealer [6]. Conventional retreatment methods that employ mechanical removal techniques using nickel-titanium (NiTi) rotary instruments have been unable to eliminate the BC sealer from the surface [6].

Recently, adjunct methods have been suggested to enhance the efficacy of removal of BC sealer, such as the use of XP-endo finisher instruments, ultrasonic-activated irrigation, and photoacoustic streaming [9–12]. Although limited to the straight area of the canal, ultrasonic tips are an excellent adjunct technique in endodontic retreatment, particularly in cases with BC sealer [13]. Ultrasonic-activated irrigation has been found to significantly increase the efficacy of sealant removal [10, 11]. In general, ultrasonic energy has been effectively employed to clean root canals from filling materials with and without BC sealer [14, 15]. However, treatment preparation with ultrasonic tips has caused a higher occurrence of microcracks [16].

In recent years, dental lasers have been advocated for a variety of uses in endodontics. Near-infrared (diode) and erbium (Er:YAg) laser with a wavelength of 2940 nm have been approved to remove the smear layer and clean and disinfect the root canal [17]. New systems applying erbium (Er:YAg) laser have been recently introduced, such as photoinduced photoacoustic streaming (PIPS) and shockwave-enhanced emission photoacoustic streaming (SWEEPS). These techniques rely on the absorption of pulses of laser energy by canal irrigants to create a series of shockwaves and turbulent photoacoustic currents, enhancing the cleaning and disinfection of the root canal [18]. Recent studies have shown that SWEEPS can enhance the antimicrobial effect of low-concentration sodium hypochlorite (NaOCl) [19]. Adjunct laser-activated irrigation has also greatly improved the removal of root-filling materials such as gutta percha and BC sealer during retreatment [10, 15, 20].

The article "Evaluation of Dentinal Microcracks following Diode Laser- and Ultrasonic-Activated Removal of Bioceramic Material during Root Canal Retreatment" was published in 2022. Journal: Scanning.

Diode laser is arguably less efficient than Er:YAg lasers due to the latter's superior absorption in water and thus canal irrigants [21]. However, diode lasers are more economical and readily available [22]. Additionally, a previous study reported that diode laser can enhance the removal of BC sealer material during root canal retreatment [15].

That said, using diode laser in root canal irrigation has been reported to decrease tooth fracture resistance [23]. Other studies have shown that microcrack creation is influenced by laser radiation in a dry canal [17, 24]. The present study is aimed at evaluating the use of microcomputed tomography (micro-CT) analysis and dentinal microcrack formation following retreatment of the BC sealer employing two adjunct techniques: ultrasonic- and laser-activated irrigation.

## 2. Materials and Methods

The randomized controlled cross-sectional in vitro study was exempt, according to Princess Nourah Bint Abdulrahman University Institutional Review Board in Riyadh, Saudi Arabia (IRB Number: 21-0435).

### 2.1. Sample Selection

For this study, thirty sound human single-canal teeth, which had been extracted for periodontal or orthodontic reasons, were selected according to predefined criteria. Teeth with calcification, open apices, abnormally short roots, visible root fractures or cracks (under magnification), root resorption or erosion, or more than one canal in the root were excluded. The teeth were preserved in saline at room temperature after calculus, and soft tissue debris were removed. G^∗^Power 3.1 software (Heinrich-Heine-University, Düsseldorf, Germany) was used to calculate the sample size. It considered an effect size of 0.35, with an estimated power of 0.90 and type I error *α* of 0.05.

### 2.2. Preparation of Teeth

All crowns were cut 2 mm above the cemento-enamel junction using a straight-fissure diamond bur to guarantee uniformity and a root length of 15–18 mm. Access to the cavity was performed using access burs. The working length was calculated by inserting a size 10 K file into the canal until it reached the apical foramen; then, 1 mm was reduced. Only teeth where the initial apical file was a size 10 or 15 K files were included. To form a closed system, the canal apex was closed with a soft piece of wax, and the tooth was lodged in silicon. All canals were prepared using ProTaper Universal files (Dentsply Maillefer, Ballaigues, Switzerland) to size F3, regularly irrigating with 2.5% NaOCl (1 mL) between each file, with a final irrigation of 17% EDTA (3 mL) and normal saline (5 mL). Before obturation, the canals were dried with paper points. The TotalFill BC sealer (FKG Dentaire SA, La Chaux-de-Fonds, Switzerland) and a single standardized gutta percha cone size F3 (Dentsply Maillefer, Ballaigues, Switzerland) were used to fill all root canals using the single-cone method. To allow for the complete setting of the BC sealer, all teeth were placed in a humidor for three weeks at 37°C and 100% relative humidity.

The article "Evaluation of Dentinal Microcracks following Diode Laser- and Ultrasonic-Activated Removal of Bioceramic Material during Root Canal Retreatment" was published in 2022. Journal: Scanning.

### 2.3. Retreatment

Mechanical retreatment was carried out using D-Race NiTi rotary instruments (FKG Dentaire SA, La Chaux-de-Fonds, Switzerland) with 20 mL of saline. The root canal filling material was removed, and patency was obtained with a size 15 K file, followed by taking a size F3 ProTaper Universal instrument to the working length. The sample (*n* = 30) was then randomly divided into three equal groups: group 1 was the control group, and group 2 underwent passive ultrasonic irrigation using a size 15 ultrasonic K file (Satelec Ultrasonic Unit) with 2.5% NaOCl followed by saline. In group 3, a laser diode (Master lase/expert lase, Kavo, Biberach/Ri*β*, Germany) with a wavelength of 980 nm, a frequency of 100 Hz (37°C), and a power of 2.5 W were used.

The protocol conducted in groups 2 and 3 was previously described for effective retreatment of BC sealer filling material [15].

Passive ultrasonic irrigation was conducted by inserting the ultrasonic file into the canal 1 mm short of the full working length. It was activated for a total of 1 min in three 20 sec cycles, with 3 mL of 2.5% NaOCl. This was repeated five times, followed by final activation for 1 min using 5 mL of saline.

For teeth in group 3, the laser diode 300 *μ*m fiber tip was introduced into the canal and activated at a distance of 1 mm from the working length for 10 secs. During every activation, the tip was gently withdrawn and then reinserted along the entire length of the root canal in a helical movement. This was repeated for a total of 1 min for every specimen with 3 mL of 2.5% NaOCl then with 5 mL of saline.

All irrigants were delivered into the canal using monovac Luer lock 30-gauge side-vented irrigation needle tips and inserted 1 mm short of the full working length.

### 2.4. Evaluation of Dentinal Defects

Using micro-CT, teeth were scanned four times: before and after root canal preparation, then after the mechanical retreatment using NiTi rotary instruments, and finally, after the use of ultrasonic and laser energy. To guarantee that teeth were scanned in the same location each time, silicone molds were made for each root. The teeth were stored in a humidor before and after each scan.

The article "Evaluation of Dentinal Microcracks following Diode Laser- and Ultrasonic-Activated Removal of Bioceramic Material during Root Canal Retreatment" was published in 2022. Journal: Scanning.

Two calibrated trained observers who were experienced endodontists viewed the cross-sectional images on Data Viewer (Skyscan, Kontich, Belgium) and calculated the number of dentinal defects according to the method described by Almeida et al. [7]. The presence of any type of defect, whether a crack or craze line on the external root surface or internal canal wall, was counted. The images from the postirrigation scans were viewed first, and the slice number associated with the defect was recorded. The same slice was then evaluated in the post retreatment and post- and preinstrumentation scans to see whether the defect was also present. Interobserver agreement calculated using the intraclass correlation coefficient was found to be 0.948, indicating excellent interobserver agreement. Cases of disagreement were analyzed by both examiners until an agreement was reached. The process was repeated after four weeks.

### 2.5. Statistical Analysis

SPSS (IBM Corp. Released 2013. IBM SPSS Statistics for Windows, Version 22.0. Armonk, NY, USA: IBM Corp.) was used to analyze the data. After the normality of the data was explored using the Shapiro–Wilk test, Friedman's two-way analysis of variance by ranks was used to compare the number of cracks pre- and posttreatment. Fisher's exact test was used to compare the percentage of cracks. The statistical significance level was set at *p* < 0.05.

## 3. Results

In total, 32,300 slices were inspected, and 11,845 slices contained cracks.  Table 1 shows the percentage of cracks pre- and posttreatment. A significant increase occurred in the number of cracks postmechanical retreatment and activated irrigation compared to both pre- and postinstrumentation (*p* = 0.0001). However, activated irrigation protocols did not result in a significant increase in the number of cracks compared to the mechanical retreatment (*p* = 0.345; Figure 1).

The coronal and middle canal thirds showed a significant increase in the number of cracks postmechanical retreatment and activated irrigation compared to pre- and postinstrumentation (*p* = 0.001). However, cracks in the apical third showed no significant change (*p* = 0.90; Figure 2).

A comparison between ultrasonic and laser irrigation revealed no significant difference between the percentage of cracks after laser and ultrasonic irrigation (*p* = 1.00).

## 4. Discussion

Nonsurgical retreatment of root canals filled using BC sealer has been deemed problematic [6, 7]. Photoacoustic techniques such as PIPS and SWEEPS can improve root canal filling removal during root canal retreatment [20]. Recently, laser- and ultrasonic-activated irrigation have been proposed as adjunct procedures to enhance the complete removal of the BC sealer material [10, 15, 25, 26]. This study evaluated the toll that these treatments may have on the dentinal root in terms of dentinal defects that jeopardize the tooth's longevity.

The article "Evaluation of Dentinal Microcracks following Diode Laser- and Ultrasonic-Activated Removal of Bioceramic Material during Root Canal Retreatment" was published in 2022. Journal: Scanning.

The results showed no crack propagation following instrumentation using NiTi rotary files, which is in accordance with many studies that have used micro-CT to evaluate crack formation [27–30]. The association between canal instrumentation and dentinal crack formation has mainly been reported by studies using root-sectioning methods that result in specimen destruction. Not only could such methods create dentinal cracks [31, 32], but it is not possible to determine how many preexisting dentinal defects were in the specimen.

On the other hand, micro-CT, the method used in this study, is a nondestructive technique that allows a three-dimensional representation of the tooth. This facilitates comparing pre- and postoperative images with preoperative specimens serving as an authentic control [30].

Some studies have used micro-CT and found that certain instrumentation systems caused more dentinal cracks to form [33, 34]. They linked their findings to differences in instrument design, taper, number, and type of movements [4, 34–36].

One reason for the different results is that some studies did not report coregistration, which allows images taken from the same specimen at different times to be overlaid in the same place so that they can be compared accurately [33, 34].

The highest percentage of dentinal cracks in this study was found after using the NiTi rotary retreatment files. This is in accordance with many studies using micro-CT that found that NiTi rotary retreatment systems were associated with an increase in dentinal crack formation [36–38]. However, other studies reported that NiTi retreatment systems did not create dentinal cracks [7, 39].

These contradictions may be explained by discrepancies in experimental methods such as scanning and reconstruction parameters, the interval at which the cross-sectional images are examined, defect interpretation criteria, and the conditions in which the samples are stored [30]. The age of the tooth itself must also be considered. Teeth from older patients have demonstrated a greater number of dentinal cracks [40].

In this study, adjunct-activated irrigation procedures, whether ultrasonic or diode laser activation, were not associated with an increase in dentinal crack formation. Previous studies [17, 41] have shown that disinfection during root canal instrumentation using constant diode laser 980 nm irradiation (employed in this study) caused significant crack formation in the apical and middle third of the canals. These studies did not carry out their investigations using micro-CT.

The article "Evaluation of Dentinal Microcracks following Diode Laser- and Ultrasonic-Activated Removal of Bioceramic Material during Root Canal Retreatment" was published in 2022. Journal: Scanning.

However, the dentinal crack formation was associated with the use of ultrasonic tips to remove fractured instruments from the middle third of the canal [42] and create root-end preparation during periapical surgery. Researchers have reported crack formation in high-frequency settings when using ultrasonic tips for root-end preparation [43]. Such procedures involve using tips instead of the files used to activate irrigation in this study. The tip application is concentrated at a certain point that is in direct contact with the dentine, which does not happen during ultrasonic irrigant activation.

Dentinal cracks have also been linked to filling techniques that put stress on the dentinal walls [44]. However, the teeth in this study were not evaluated after root canal filling because it used the single-cone technique, which does not create such stresses and so may not initiate or propagate dentinal cracks [45].

Previous studies [36, 46] have reported an increase in crack formation focused in the apical or middle thirds [47]. In the current study, this increase was observed in the middle and coronal thirds, and not the apical third. One explanation could be related to the differences in the NiTi files used in those studies, regarding their design, mode of movement, and rotation speed [47]. Another possible explanation is the different types of teeth used in the studies. While mesial roots of molars and mandibular incisors were used in those studies [36, 46], premolars were chosen for the present study. Their canals tend to be more oval, concentrating instrumentation stresses in the middle and coronal canal thirds [47].

An important limitation of this study is that it was conducted in vitro on extracted teeth with the absence of a periodontal ligament, which would have acted as an energy absorber. Therefore, the study may have overestimated crack formation.

## 5. Conclusion

Applying laser- or ultrasonic-activated irrigation as adjunct retreatment techniques did not reveal a significant increase in dentinal microcracks in the roots. However, using NiTi rotary retreatment instruments was associated with a significant increase in dentinal microcracks. These cracks were more frequently observed in the coronal and middle canal thirds.

## Figures and Tables

**Figure 1:** Friedman's two-way analysis of variance by ranks of dentinal microcracks observed before and following mechanical and activated irrigation retreatment procedures.

The article "Evaluation of Dentinal Microcracks following Diode Laser- and Ultrasonic-Activated Removal of Bioceramic Material during Root Canal Retreatment" was published in 2022. Journal: Scanning.

**Figure 2:** Micro-CT shows the crack formation and propagation in the same slice at four different timings using laser or ultrasonic irrigation.

**Table 1:** Percentage of dentinal defects before and after retreatment procedures.

Irrigation protocol	Percentage of cracks %			
	Preinstrumentation	Postinstrumentation	Postmechanical retreatment	Postirrigation protocol
Control	13.88	13.90	49.30	49.90
Ultrasonic	33.76	55.08	68.88	68.95
Laser	0.01	0.33	53.60	57.50

## Data Availability

The datasets generated and/or analyzed during the current study are available as a supplementary file.

## Supplementary Materials

Supplementary Materials See Figure S1 in the Supplementary Material for whole dataset.
